The article "Research on Online Rapid Sorting Method of Waste Textiles Based on Near-Infrared Spectroscopy and Generative Adversity Network" was retracted in 2023. Reasons: signs of a paper mill; suspected computer-generated content; unreliable results or conclusions; concerns about the data.

# Research on Online Rapid Sorting Method of Waste Textiles Based on Near-Infrared Spectroscopy and Generative Adversity Network

**DOI:** 10.1155/2022/6215101

**Published:** 2022-05-14

**Authors:** Jinquan Hu, Huihua Yang, Guoliang Zhao, Ruizhi Zhou

**Affiliations:** ^1^School of Artificial Intelligence, Beijing University of Posts and Telecommunications, 10 Xitucheng Road, Haidian District, Beijing, China; ^2^School of Electronic Engineering and Automation Chemistry, Guilin University of Electronic Technology, No. 1 Jinji Road, Qixing District, Guilin, Guangxi, China; ^3^School of Computer Science and Information Security, Guilin University of Electronic Technology, No. 1 Jinji Road, Qixing District, Guilin, Guangxi, China; ^4^Beijing Institute of Fashion Technology, Beijing 100029, China; ^5^Shanghai Jicai Environmental Protection Technology Co., Ltd., Shanghai, China

## Abstract

In this paper, aiming at the application of online rapid sorting of waste textiles, a large number of effective high-content blending data are generated by using generative adversity network to deeply mine the combination relationship of blending spectra, and A BEGAN-RBF-SVM classification model is constructed by compensating the imbalance of negative samples in the data set. Various experiments show that the model can effectively extract the spectrum of pure textile samples. The classification model has high robustness and high speed, reaches the performance of similar products in the world, and has a broad application market.

## 1. Introduction

With the rapid development of economy and the improvement of people's daily consumption level, China consumes about 60 million tons of textiles made of various fiber raw materials every year on average [1, 2]. According to the Annual Report on Comprehensive Utilization of Resources in China published by the National Development and Reform Commission, China produces more than 25 million tons of waste textiles every year. The comprehensive utilization of waste textiles is less than 5 million tons, and the recycling rate is less than 20%. Therefore, the recycling of waste textiles is very necessary. However, due to the great difference in the component content of waste textiles, it is very difficult to screen the raw materials in the process of recycling. At present, sorting is still mainly done manually, with slow speed and low recognition rate. It cannot meet the requirements of industrial-scale production. Therefore, online efficient identification and automatic sorting at the recycling site is an important prerequisite and guarantee for the recycling of waste textiles.

The research of artificial neural network is an important branch in the field of artificial intelligence. Since Hinton put forward the deep neural network in 2006, the neural network has made great achievements in the field of information processing such as voice, image, and text [3–5]. Researchers in major universities and research institutions all over the world have vigorously carried out relevant research and proposed a variety of deep neural networks, which has greatly expanded the application of deep neural network [6, 7]. Modern deep neural network model mainly includes three basic structures: sequence-to-sequence neural network, convolution neural network, and adversarial generation network [8, 9].

Near-infrared spectroscopy (NIR) is a comprehensive technology that integrates spectral measurement technology, chemometrics, and computer technology. It is the best choice to achieve real-time, rapid, and nondestructive measurement [10]. Its online technology has been successfully applied in the fields of medicine, petrochemical, food, and agriculture, and textile testing is beginning to move from the laboratory stage to the industrial application stage [11]. The industrial application of the near-infrared spectroscopy analysis method for waste textiles is different from the laboratory mainly because of the diversity of recovered samples. For the industrial scene, the spectrum of textiles is affected by many factors such as dyeing, weaving, processing technology, damage degree, complex blending composition, and so on [12], so it is difficult to establish a complete data set. Field analysis results are much lower than laboratory results. In this paper, the deep learning method is used to deeply mine the potential distribution information of the original spectral data, and the generative adversity network is used to construct the virtual data set to compensate for the imbalance of the original data set. The test results show that the method can effectively improve the completeness of the data set and the accuracy of the model.

## 2. Experimental Part

### 2.1. Experimental Instruments

In this paper, the noncontact diffuse reflectance near-infrared spectrometer DA7440 of Pertern Company was used as the spectrum acquisition equipment, the spectral range was 950∼1650 nm, the resolution was 5 nm, the number of scans was 100, and the time to generate the spectrum was less than 700 millisecond.

### 2.2. Source of Samples

All samples, collection equipment, and experimental sites are provided by Shanghai JICAI Environmental Protection Technology Co., Ltd., and the chemical analysis results (labels) of the samples are provided by the Beijing Institute of Fashion Technology. Since the most valuable part of the recycled waste textiles is the pure textiles of various materials, the sample set is shown in Table 1.

The pure material samples and the blended samples in the table are divided into a training set and a test set according to different proportions and are used for training the model. The field test set is used for the final performance verification and evaluation of the model. The field test included 3 pieces of pure acrylic, 48 pieces of pure cotton, 47 pieces of pure polyester, 41 pieces of wool, and 86 pieces of blended yarn.

### 2.3. Sample Set Characteristics

Recycled waste textiles are usually used and idle for several years, with various varieties and colors, unknown processing conditions, different degrees of damage, different thicknesses, and random spectral acquisition positions, and are easily affected by buttons and zippers, which lead to different degrees of spectral changes and affect the classification performance of the model.

Figure 1 shows a raw near-infrared spectrum of a portion of a textile.  Figure 1(a) shows two spectra of pure acrylic, pure cotton, pure polyester, and pure wool samples, respectively. It can be seen that different kinds of pure materials have their own characteristics, and there are great differences between them. It is easy to distinguish different pure materials. However, it also shows that it is difficult to obtain good classification performance if the pure material samples are used as the positive and negative samples of the training model, respectively.  Figure 1(b) is the original spectrum of some pure wool, which shows that pure wool samples have some common characteristics, but some samples show obvious other characteristics because the sample label does not contain the color, process, and other information of the sample. It is not possible to determine the specific reasons for the different characteristics of the same material sample, but the model must be able to accurately extract the pure material samples affected by various factors.  Figure 1(c) shows the spectra of some pure wool and wool-containing blended samples. It can be seen that different contents, different material blends, and blending processes will have different degrees of impact on the spectra of samples. High content of blended samples and some special blended samples (such as viscose) will seriously affect the classification accuracy of the model, and these samples will be better as the negative samples of the training model. But in fact, there are many kinds of blended fabrics, and it takes a lot of time and economic cost to get more blended samples.  Figure 1(d) shows the spectra of some pure cotton samples with different colors. It can be seen that different color processes will have a great impact on the spectrum of the sample. Of course, in addition to the different colors of these samples, it is uncertain whether other processing processes are the same, so it is uncertain whether the impact is entirely caused by dyeing, but it can be explained that for waste textiles, many factors will cause great changes in the spectrum of samples, thereby increasing the classification difficulty of the model.

In general, the near-infrared spectra of waste textiles have obvious species characteristics, but they are also affected by many factors, and the samples that cause classification errors are mainly some high-content blends and some special process blends. Collecting more data sets is the best way to improve the accuracy of the model, but it takes a lot of time and economic costs. It is very difficult for the industry to work after obtaining a complete data set, and we must deal with these problems as much as possible from the algorithm.

## 3. Algorithm Structure

The research on the application of near-infrared spectroscopy in textile classification and quantitative analysis has been widely carried out in various research institutions and universities, and many mature algorithms have been accumulated. However, most of the algorithms are aimed at some specific applications or specific types of processing methods, and there are few comprehensive application methods for all waste textiles. There is still a large research gap in the field of industrial application. Because the composition information of textiles needs to be determined by chemical methods, the cost of time and economy is relatively high, resulting in a small number of data sets and unbalanced distribution, which greatly affects the performance of the model. One way to deal with data imbalances is to create virtual data sets. The generative adversarial network (GAN) [13–15] has an excellent performance in this respect. In this paper, the virtual blending data set is constructed by using the generative antagonistic network structure to supplement and improve the blending data, especially the high content blending data, so as to provide the accuracy of classification and other performances.

The GAN was first created by Ian Goodfellow in 2014 and consists of a generator (*G*) and a discriminator (*D*), both of which are multilayer perceptual networks, as shown in Figure 2. The generator fabricates data from a random noise *Z* input, and the discriminator is responsible for determining whether the data are true and giving a score.

The objective function of the GAN model is represented by the following:

(1) $$\begin{array}{c} \underset{G}{\min}\underset{D}{\max}V\left(D,G\right)=E_{x∼p_{\text{data}\left(x\right)}}\left[\log D\left(x\right)\right]+E_{z∼p_{\text{data}\left(z\right)}}\left[\log\left(1-D\left(G\left(z\right)\right)\right)\right]. \end{array}$$

The log [*D* (*x*)] in the first item represents the result of the discriminator's judgment of the real data, and the second item represents the synthesis and judgment of the data. The generators and discriminators are trained alternately through a two-sided game between the maximum and minimum values until the Nash balance is reached. Given any generator *G*, the training criteria for discriminator *D* are to maximize *V* (*D*, *G*). Therefore, assuming that the generator is fixed, the maximized objective function can be represented by the following formula:

(2) $$\begin{array}{c} V\left(D,G\right)=\int_{x}p_{\text{data}}\left(x\right)\log\left(D\left(x\right)\right)+p_{g}\left(x\right)\log\left(1-D\left(x\right)\right)\text{d}x. \end{array}$$

The formula for calculating the optimal discriminator is

(3) $$\begin{array}{c} D_{G}^{*}\left(x\right)=\frac{p_{\text{data}}\left(x\right)}{p_{\text{data}}\left(x\right)+p_{g}\left(x\right)}. \end{array}$$

The optimal discriminator is substituted into the objective function *V* (*D*, *G*) to obtain the objective function of *G*:

(4) $$\begin{array}{c} C\left(G\right)=E_{x∼p_{\text{data}}}\left[\log\frac{p_{\text{data}}\left(x\right)}{p_{\text{data}}\left(x\right)+p_{g}\left(x\right)}\right]+E_{x∼p_{g}}\left[\log\frac{p_{g}\left(x\right)}{p_{\text{data}}\left(x\right)+p_{g}\left(x\right)}\right]. \end{array}$$

When *p*_*g*_=*p*_data_, *D* = 0.5, the discriminator cannot distinguish between real samples and generated samples, and the generator perfectly replicates the data generation process.

In this paper, Boundary Equilibrium GAN (BEGAN) is used. The optimization objective of BEGAN is slightly different from that of the original GAN. BEGAN requires that the reconstruction error distribution of the two should be as close as possible. The reconstruction error is calculated by

(5) $$\begin{array}{c} L\left(v\right)={\left|v-D\left(v\right)\right|}^{\eta }, \end{array}$$

where *V* represents the input data of the discriminator; *D* (*V*) represents the output of the discriminator *D*, and *η* is the norm selection parameter.

BEGAN uses proportional control theory during training to keep the balance between the generator and the discriminator during training, namely

(6) $$\begin{array}{c} \gamma =\frac{E\left[L\left(G\left(z\right)\right)\right]}{E\left[L\left(x\right)\right]}. \end{array}$$

When training, you can choose *γ* to adjust the generation effect. Proportional control theory makes the training stable and fast and greatly improves the convergence speed of the network.

The network structure of the system is shown in Figure 3. The whole network structure is composed of a generator *G*, a classifier *C*, and a discriminator *D*, wherein the generator *G* and the discriminator *D* are multilayer perceptrons, and the classifier *C* is a pretrained Gaussian kernel support vector machine. The inputs *I*1 and *I*2 of the generator *G* are two randomly selected pure material spectra, and Z is a random number. *I*pred is the output of the generator. It is the mixture spectrum of *I*1 and *I*2 generated by simulation, and the mixture ratio is randomly selected between 50% and 99%. The discriminator uses the error between the output Ipred of the Wasserstein distance metric generator and the mixed material spectrum i3 and ends the training when the two are balanced. The optimization objectives of the discriminator and the generator are

(7) $$\begin{array}{c} L_{D}=L\left(I3\right)-k_{t}L\left(I\text{pred}\right),\\ L_{G}=L\left(I\text{pred}\right),\\ k_{t+1}=k_{t}+\lambda_{k}\left[\gamma L\left(x\right)-L\left(G\left(z\right)\right)\right]. \end{array}$$

The classifier *C* is trained with the pure material spectrum *I*4 as a positive sample in advance so that it has the ability to correctly classify the pure material spectrum. The classifier uses the output *I*pred of the generator as a negative sample to ensure the diversity of *I*pred in the training process of the antagonistic network.

## 4. Experiment and Analysis

In order to test the effectiveness of the algorithm, several experiments are carried out. The first experiment is the spectrum generation experiment, which is used to verify that the generative antagonistic network can effectively generate the mixed sample spectrum. The second experiment is the classification model training and testing experiment, which compares the performance of the classification model with other classification models. The third experiment is a field test experiment, in which the classification model is deployed in the sorting system, and the operators test the accuracy and classification time on the spot.

### 4.1. Spectrum Generation Experiment

Experimental environment: CPU: Intel Core I9, memory: 32 GB, GPU: Nvidia GT1080, operating system: WIN10, software: PYTHON.

Experimental method: After the training of the generated antagonistic network, take several outputs of the generated network, record the mixing parameters, and draw the spectrum as shown in Figure 4.

Figure 4(a) shows part of the generated spectrum and part of the actual spectrum. There is no connection between them, but it can be seen that they all reflect the peak characteristics of the main components.  Figure 4(b) shows two selected spectra with close mixing ratios, in which the first and third spectra are generated spectra, and the second and fourth spectra are actual spectra. It can be seen that the generated spectrum not only reflects the peak characteristics of the main components but also reflects the diversity, which can enrich the spectral samples of blended materials and improve the classification performance.

### 4.2. Comparison Experiment of Classifier Performance

The experimental environment is the same as above.

Experimental method: The data set shown in Table 1 was used for the experimental data set, and the first derivative of SG and SNV was used for the spectral preprocessing method. Firstly, all pure material spectrum samples are used to train RBF-SVM, then all blended samples are used to train BEGAN, and then 1000 50%–99% random component mixed spectra are generated by the trained generator as negative samples. Finally, all the pure material spectra, blended spectra, and the generated spectra were used to synthesize the data set, which was divided into training set and test set according to the ratio of 9 : 1, and RBF-SVM was trained and tested by grid optimization method. The comparison algorithms include linear SVM, extreme learning machine, KNN, and decision tree. The training set and test set are allocated by leave-one-out method, and the average value is obtained by repeating 50 times. Considering the imbalance of positive and negative samples, this paper uses sensitivity and specificity to measure the performance of each classifier, and the experimental results are shown in Table 2:

It can be seen from the above table that the performance of various conventional machine learning algorithms is relatively close, among which the effect of KNN is slightly better, but its decision time for a single sample is much longer than that of other algorithms, and the test time on the local machine is more than 300 ms per sample, which is not suitable for on-site rapid measurement. It should be noted that although the algorithm in this paper has obvious advantages, it can only show that the algorithm can effectively classify but cannot fully explain its superiority over other algorithms because they do not use the same training set and test set. It should also be noted that the specificity for acrylic is 0 because there is only one sample with more than 50% acrylic in the blend sample.

The one-class SVM algorithm in the above table is a classification algorithm designed for unbalanced data sets. This method only uses the original data sets for training and testing. It can be seen from the results in the table that the performance of this method is close to that of other traditional methods and slightly inferior to that of the algorithm in this paper.

### 4.3. Classifier Field Accuracy Test Experiment

Experimental environment: The sorting system uses a desktop computer as the main controller, the CPU is Intel Core i7, the memory is 16 GB, and there is no GPU. The computer is connected to the near-infrared spectrometer DA7440 of Pertern Company through the network interface, and it takes 0.9 seconds to collect one spectrum and generate a CSV file. The algorithm is deployed in the WINDOWS application, and the trained model is used to complete the classification by reading the data in the CSV file.

Experimental method: 225 pieces of waste clothes with tags are provided on-site and placed on the sorting line one by one by the operator. The sorting line is equipped with a weighing sensor as the starting valve for starting a sorting. The schematic diagram of the sorting line is shown in Figure 5. When the weighing sensor detects the textile, it will delay 200 ms to start the spectrometer to collect the spectrum, and then control the turntable system to put the textile into the corresponding box after spectrum preprocessing and classifier judgment.

Because each part works in parallel, the average processing time of each textile is less than 1.2 seconds and meets the sorting requirements of 2000 pieces per minute. When 225 test samples were sorted, the operator manually counts the sorting results according to the sorting results of each sample and the tag on it and repeats three times. The test results are shown in the following table.

In the above table, TP represents the positive sample of correct prediction, that is, the high-value sample to be extracted, which should be as close as possible to the actual number. FP indicates the positive sample of error prediction, that is, the blended sample is judged to be a pure material sample, which is a misjudgment and will reduce the purity of the product. At present, the purity of recycled waste textiles in the market is 93%–95%. The average accuracy rate of the above table is higher than the average level of the market, which fully meets the quality requirements. FN indicates the positive sample of wrong prediction, that is, the pure material sample is judged as the blended sample, which is a missed judgment and will reduce the benefit of the product. The average recall rate in the above table basically meets the benefit requirements of industrial production.

It should be noted that the test results in the above table are better than the results of Experiment 2, which is not consistent with the general industrial situation. This is because in most of the recycled waste blended samples, the proportion of each content is in the range of 3/7, 2/8, or 4/6, and the proportion of 90% or even more than 95% is less. In the training process of the model, many high-content blended samples are generated as negative samples, so the model generally does not misjudge the low-content blended samples. The reason for missing judgment may be that the position of spectrum acquisition is affected by other factors such as too thin textile, zipper or button, and special dyeing process, which causes great changes in the spectrum.

In particular, the data set was manually sorted by several workers before being sent to the laboratory for chemical composition analysis. Then, according to the results of the chemical composition analysis, the sorting accuracy is between 50% and 80%, which is related to the proficiency of workers and the sorting speed. After the chemical analysis of the sample, the component label is nailed on the collar. Considering the memory ability of workers, the comparison test with manual sorting will not be carried out after the sorting equipment is adopted.

### 4.4. Field Batch Pure Material Spectrum Extraction Experiment

The experimental environment is the same as above.

Experimental method: The pure material samples on the spot were mixed into 3000 unknown samples, then sorted by the sorting line, and then, the operator manually searched and compared the classification results of these pure material samples and repeated three times, and the test results are shown in the following table.

Since the situation of 3000 unknown samples is unknown, it is impossible to judge whether there is a misjudgment (blended yarn is judged as pure yarn), and only the TP and FN values of pure yarn samples with tag labels are counted. Compared with the results in Table 3, the results in Table 4 do not decrease significantly, indicating that the system model has high robustness and is fully suitable for industrial application.

## 5. Conclusion

In this paper, aiming at the current situation of waste textile recycling at home and abroad, this paper puts forward an online rapid sorting application method based on near-infrared spectroscopy. Recycling enterprises are limited by the scale of economic investment, it is difficult to build a complete textile near-infrared spectrum analysis data set, and the effect of using traditional near-infrared spectrum analysis methods is poor. In this paper, the combination relationship of the blending spectrum is deeply mined by generating countermeasure network, a large number of effective high content blending data are generated, the negative sample imbalance of the data set is compensated, and the BEGAN-RBF-SVM classification model is constructed. Various experiments show that the model can effectively extract the spectrum of pure textile samples. The classification model has high robustness and fast speed, which reaches the performance of similar international products and has a broad application market.

## Figures and Tables

**Figure 1:** Several original spectrograms.

**Figure 2:** Generative adversarial network.

**Figure 3:** Schematic diagram of overall network structure.

**Figure 4:** Generated spectrogram.

**Figure 5:** Schematic diagram of sorting line.

**Table 1:** Sample type and quantity.

Serial number	Species	Quantity
1	Pure acrylic fiber	75
2	Pure cotton	226
3	Pure polyester	240
4	Pure wool	473
5	Blending	100
6	Pure viscose fiber	1
7	Pure silk	1
8	Field test set	225

**Table 2:** Comparison of classifier performance.

Performance	CLASS	BEGAN-RBF-SVM	Linear-SVM	ELM	KNN	Precision Tree	One-class SVM
Sensitivity	Acrylic	0.97	0.91	0.90	0.94	0.88	0.92
	Cotton	0.94	0.89	0.89	0.91	0.85	0.88
	Poly	0.94	0.90	0.91	0.92	0.83	0.90
	Wool	0.93	0.85	0.83	0.87	0.82	0.87

Specificity	Acrylic	0.01	0	0	0	0	0
	Cotton	0.05	0.13	0.12	0.08	0.16	0.15
	Poly	0.06	0.09	0.13	0.05	0.11	0.10
	Wool	0.08	0.16	0.15	0.04	0.23	0.17

**Table 3:** Experimental results of on-site classification accuracy test.

Times	Category	Actual quantity	TP	FP	FN	Accuracy (%)	Recall (%)	Average accuracy (%)	Average recall (%)
1	Acrylic	3	3	0	0	100	100	100	100
	Cotton	48	47	0	1	100	98	100	98.7
	Poly	47	46	0	1	100	97.9	100	97.9
	Wool	41	41	2	0	95.3	100	96.1	98.4
	Others	86							

2	Acrylic	3	3	0	0	100	100		
	Cotton	48	48	0	0	100	100		
	Poly	47	46	0	1	100	97.9		
	Wool	41	40	1	1	97.6	97.6		
	Others	86							

3	Acrylic	3	3	0	0	100	100		
	Cotton	48	47	0	1	100	98		
	Poly	47	46	0	1	100	97.9		
	Wool	41	40	2	1	95.3	97.6		
	Others	86							

**Table 4:** Experimental results of field batch pure material sample extraction.

Times	Category	Actual quantity	TP	FN	Recall (%)	Average recall (%)
1	Acrylic	3	3	0	100	100
	Cotton	48	46	2	95.8	98.6
	Poly	47	46	1	97.9	97.9
	Wool	41	40	1	97.6	98.4
	Others	3000				

2	Acrylic	3	3	0	100	
	Cotton	48	48	0	100	
	Poly	47	47	0	100	
	Wool	41	40	1	97.6	
	Others	3000				

3	Acrylic	3	3	0	100	
	Cotton	48	48	0	100	
	Poly	47	45	2	95.7	
	Wool	41	41	0	100	
	Others	3000				

## Data Availability

No data were used to support this study.
